RETRACTED

# Assessment of nitrogen-fixing endophytic and mineral solubilizing rhizospheric bacteria as multifunctional microbial consortium for growth promotion of wheat and wild wheat relative *Aegilops kotschyi*^☆^

**DOI:** 10.1016/j.heliyon.2022.e12579

**Published:** 2022-12-25

**Authors:** Rajeshwari Negi, Tanvir Kaur, Rubee Devi, Divjot Kour, Ajar Nath Yadav

**Affiliations:** a Microbial Biotechnology Laboratory, Department of Biotechnology, Dr. Khem Singh Gill Akal College of Agriculture, Eternal University, Baru Sahib, Sirmour, 173101, Himachal Pradesh, India; b Department of Microbiology, Akal College of Basic Sciences, Eternal University, Baru Sahib, Sirmour, 173101, Himachal Pradesh, India

**Keywords:** Agricultural sustainability, *Aegilops kotschyi*, Bioinoculants, Endophytes, Wheat, Plant growth promotion

## Abstract

Microbes play crucial functions in maintaining the health and growth of the plants directly or indirectly by supplying nutrients. These microbes could be used as biofertilizers for the enhancement of soil health and growth of crops. In preset investigation, potential microbes from endophytic and rhizospheric region of *Aegilops kotschyi* growing in green slopes of Shivaliks, Himachal Pradesh were sorted out and screened for plant growth promoting attributes including phosphorus and potassium solubilization. The potential bacterial strains were identified through 16S rRNA gene sequencing and developed as microbial consortium for the plant growth of wheat and wild wheat relative *Aegilops kotschyi*. A total 125 isolates of bacteria were sorted out and among them 36 were found as P-solubilizers and 19 showed K-solubilization attribute and two highly potential bacterial strain were identified as *Bacillus tropicus* EU-ARP-44 (P-solubilizer; 270.5 ± 0.00 mg L^−1^) and *B. megaterium* EU-ARK-23 (K-Solubilizer; 51.3 ± 1.7 mg mL^−1^). The microbial consortium of *Rahnella* sp. strain EU-A3SNfb (N-fixer; MN294545), *B. tropicus* EU-ARP-44 (P-solubilizer) and *B. megaterium* EU-ARK-23 (K-solubilizer) evaluation in *Aegilops kotschyi* and wheat crop resulted in the enhancement of growth as well as physiological parameter including shoot/root length, fresh/dry weight and chlorophyll, carotenoid, total soluble sugar content, phenolic and flavonoid content as compared to un-inoculated control. Microbial consortium consisting of potential plant growth promoting (PGP) bacterial strains could be used as biofertilizer and bioinoculants in cereals crop growing in hilly region.

## 1 Introduction

Cerealis derivative ‘cereals’ are a type of grasses that are consumed all over the globe as it provide much more energy than any other crop type. They are rich sources of minerals, carbohydrates, vitamins, fats, proteins and oils. Worldwide different types of cereals are grown such as rice, millet, wheat, sorghum, barley, rye and maize (Muhammad et al., 2013). Wheat (*Triticum aestivum*) is one of the oldest and important cultivable staple crop of the globe as it forms cohesive dough that could be made into noodles, soup, pasta and other food products. The appropriate production of wheat requires a huge amount of macronutrients including phosphorus (P), nitrogen (N) and potassium (K) which are the most essential requirement for the production of wheat. The nutrient NPK helps in the uptake and assimilation of other nutrients, protein biosynthesis, biomass production and yield. The amount of available form of nutrients (NPK) is fewer in soil and insufficient supply may leads to reduced wheat yield. To fulfill the nutrient requirement, externally NPK fertilizers were being added throughout the world which helps in increasing the wheat yield. The external fertilizers added usually developed through the chemical processes and they are known to leave a deleterious effect on the environment, humans, animals, and soil macro and microflora.

RETRACTED

Beneficial microbes associated with plants could be used in agricultural farms as an alternative of chemical fertilizers. Plant associated microflora plays significant role in improving soil fertility, plant health and growth (Jyolsna et al., 2021; Yadav et al., 2021). Apart from plant growth promotion, and soil fertility, plant and soil microbiomes plays a vital role in agricultural sustainability (Devi et al., 2022a). Beneficial microbes such as fungi, bacteria, and archaea exist in diverse habitats such as plant (endophytic, phyllospheric, and rhizospheric), soil, and water (Doty 2017b). Microbes serve a crucial function in maintaining the health and growth of plant directly or indirectly by supplying nutrients, such as N, P, K, Fe and Zn and producing secondary metabolites and ammonia that are antagonistic to pathogenic microbes (Sylia et al., 2022; Verma et al., 2015, 2016). These microbes also helps in protecting plants from various abiotic stress factors such as drought tolerance, high/low temperature, low/high pH, the presence of heavy metals, and high salinity (Verma et al., 2016; Sharma et al., 2021).

Unfortunately, despite the fact plant–microbe interaction is beneficial; it was often overlooked for longer period of time (Smith et al., 1999). Now day's microbes are used as bioinoculants and they are applied as single inoculum and microbial consortium (Devi et al., 2022c; Kaur et al., 2022). Microbial blend of microbes i.e. microbial consortium is a better bioinoculant as it helps in the enhancing the crop productivity more efficiently in comparison with single culture containing bioinoculant. In a report, the microbial mixture of *Bacillus subtilis* and *Trichoderma harzianum* significantly incremented the growth parameters and yield in tomato plant as compared to singly inoculated bacteria (Kumar et al., 2015). In the present investigation endophytic and rhizospheric bacteria associated with wild variety of wheat namely, *Aegilops kotschyi* were isolated, characterized for phosphorus and potassium solubilization; and microbial consortium was developed and evaluated on *Aegilops kotschyi* and wheat under both *in vitro* and *in vivo* conditions.

RETRACTED

## 2 Materials and methods

### 2.1 Sampling area and isolation of bacteria from *Aegilops kotschyi*

The rhizospheric soil, and plant of *Aegilops kotschyi* were collected from the Himalayan mountains on the green slopes of the Shivaliks (30.7537° N, 77.2965° E), Himachal Pradesh in clean plastic bags and stored at 4 °C temperature until isolation. The isolation of culturable endophytic and rhizospheric bacteria were performed using serial dilution plating technique on various selective and non-selective growth media including King's B agar, T_3_A agar, nutrient agar (NA), tryptic soy agar and ammonium mineral salt (AMS) (Verma et al., 2015; Kour et al., 2020). The isolation was further followed by the bacterial culture purification (on respective growth media) and preservation (nutrient agar slants and 25% glycerol stock).

### 2.2 Screening of bacteria for phosphorus and potassium solubilization

***Phosphorus solubilization***: The qualitative estimation of P-solubilization was done onto Pikovskaya agar medium supplemented with 0.5% insoluble form of P (apatite, rock phosphate and tricalcium phosphate) through spotting method (Pikovskaya 1948). The inoculated plates were incubated in the BOD incubator at 28 °C for 5–7 days for the clear zones formation. The bacterial strains showing P-solubilization activity onto Pikovskaya agar plates were subjected to quantitative estimation of P-solubilization. The quantitative estimation was done by inoculating 1 mL of culture in 25 mL of 0.5% tricalcium phosphate amended Pikovskaya broth. After the incubation of 7 days, the suspensions of the isolates were centrifuged (15 min; 10,000 g) and supernatant optical density (OD) was estimated at 600 nm. The P concentration was expressed in mg L^−1^ (Murphy and Riley 1962).

***Potassium solubilization***: Potassium solubilizing ability of bacterial were qualitatively and quantitatively estimated accordingly Hu et al. (2006) and Sugumaran and Janarthanam (2007), respectively. Qualitative estimation of K-solubilization was carried out onto Aleksandrov's agar amended with mica (0.2%) as sole source of K. The inoculated plates with selected bacterial strains were kept in BOD incubator for 5–7 days at 28 °C. The bacterial cultures forming clear zone were further used to quantitative estimation of K-solubilization. The quantitatively K-solubilization was estimated by inoculating bacterial isolates in 0.2% mica supplemented Aleksandrov's broth (50 mL). After the 7 day of incubation (150 rpm and 28 °C) the suspension of isolates were centrifuged (10,000 rpm; 10 min) and content of K in the supernatant was estimated using flame spectrophotometry. The K concentration was expressed in mg mL^−1^.

RETRACTED

### 2.3 Identification and phylogenetic analysis of selected NPK bacterial strains

The selected bacterial strains were molecularly identified using gDNA isolation and 16S rRNA gene amplification. The genomic DNA (gDNA) of the selected NPK bacterial strains were isolated as per the method described by Yadav et al. (2015). Afterwards, isolated gDNA of bacterial strains were subjected to 16S rRNA gene amplification using pA and pH primers to obtain fragment (nearly 1540-bp). Afterwards purification of amplified products of PCR using QIA quick purification kit (Qiagen) and sequencing was done from Xcelris lab Ltd., Ahmedabad. The bacterial strains were identified using BLASTn program in NCBI. The phylogenetic tree was constructed using program MEGA 4.0.2. through neighbor joining method (Tamura et al., 2007).

### 2.4 Development of bacterial consortium

The bacterial consortium of N-fixer, P- and K-solubilizer was prepared using three potential strains of bacteria i.e. *Rahnella* sp. strain EU-A3SNfb (N-fixer; MN294545) isolated previously (Negi et al., 2022), EU-ARP-44 (P-solubilizer), and EU-ARK-23 (K-solubilizer). The selected efficient bacterial isolates were assessed for their compatibility using cross streaked assay onto nutrient agar medium and developed as consortium according to method of Kaur et al. (2022). Afterwards the cultures growth, colony-forming units (CFU) was calculated. The culture media of three bacterial cultures were mixed in an equivalent amount and the bacterial consortium was developed for further evaluation.

### 2.5 Evaluation of bacterial consortium

The individual and microbial consortium effect of three potential strains i.e. *Rahnella* sp. strain EU-A3SNfb (1.23 × 10^7^ CFU mL^−1^), EU-ARP-44 (3.46 × 10^7^ CFU mL^−1^), and EU-ARK-23 (2.90 × 10^7^ CFU mL^−1^) exhibiting N-fixation, P-solubilization, and K-solubilization attributes, respectively were evaluated for the growth promotion of *Aegilops kotschyi* and wheat under both *in vitro* and *in vivo* conditions. The experiment was carried out during the month of November 2021 to April 2022 with total eight treatments viz. T1 (bacterial consortium); T2 (EU-A3SNfb); T3 (EU-ARP-44); T4 (EU-ARK-23**);** T5 (recommended dose of NPK); T6 (recommended dose of urea); T7 (recommended dose of di-ammonium phosphate); and T8 (control) and all replicated three times in both *in vitro* and *in vivo* conditions. The *in vitro* evaluation of bacterial consortium in *Aegilops kotschyi* and wheat was carried out in 4 kg non-sterile soil (pH 6.9, available N 390 kg ha^−1^, available P 15.3 kg ha^−1^, available K 212 kg ha^−1^, organic carbon 0.65%, and iron 12 mg kg^−1^) filled in plastic pots of size 30 cm × 30 cm × 26 cm and all pots were distanced equally from each other to reduce the cross contamination. In each plastic pot, six bacterized seeds were sown and after the seed germination four plants were maintained till the harvesting. The *in vivo* evaluation of bacterial consortium was conducted at the Experimental Farm, Machher (30.7537 N, 77.2965 E), Eternal University, Baru Sahib, District Sirmour, Himachal Pradesh, India. The field randomized block design was followed. The seeds of *Aegilops kotschyi* and wheat were coated with sugar solution and treated with cultures (single inoculum and bacterial consortium) in ration of 1:1 before the sowing. After the 90 days of sowing, growth and physiological parameters of both *Aegilops kotschyi* and wheat were recorded.

RETRACTED

### 2.6 Examination of growth and physiological parameters

The growth parameters including fresh/dry biomass, length, of shoot/root were studied at 90 days of sowing. The chlorophyll and carotenoid content was estimated as per method described by Lichtenthaler (1987). The determination of phenolics and flavonoids content in pearl millet leaf were done as per earlier described method of Kim et al. (2003) and Park et al. (2008), respectively. *Aegilops kotschyi* and wheat total soluble sugar content was performed as per the method of Irigoyen et al. (1992).

### 2.7 Statistical analysis

The obtained data was subjected to Student's t-test statistical significance. Mean comparisons were conducted using the critical difference (5%) and least significant difference (LSD) test (P = 0.05). LSD and standard error results were calculated.

## 3 Results

### 3.1 Sampling area and isolation of endophytic and rhizospheric bacteria

Endophytic and rhizospheric bacteria from different crops cultivated in Baru Sahib, Himachal Pradesh were isolated on different growth medium. A total 125 endophytic and rhizospheric bacteria were isolated from different crops. Population of bacterial isolates varied from 0.44×10^7^ to 4.16 × 10^7^ CFU g^−1^ of sample. The maximum bacterial diversity was supported on NA medium and least population was supported by AMS for both rhizospheric soil and plant samples.

RETRACTED

### 3.2 Screening of bacteria for phosphorus and potassium solubilization

Among 125 bacteria, thirty six strains were able to solubilize P ranging from 111.0 ± 0.03 mg L^−1^ to 270.5 ± 0.00 mg L^−1^ and nineteen isolates were having ability of K-solubilization ranging from 5.11 ± 0.05 mg mL^−1^ to 51.3 ± 1.7 mg mL^−1^. Among P- and K-solubilizer strain EU-ARP-44 solubilized highest P (270.5 ± 0.00 mg L^−1^) and EU-ARK-23 (51.3 ± 1.7 mg mL^−1^) solubilized highest potassium.

### 3.3 Identification and phylogenetic analysis of selected NPK bacterial strains

The partial sequences of bacterial strains (16S rRNA gene) achieved afterwards sequencing were compared using BLASTn algorithm with those sequence present in NCBI database. The BLASTn analysis of two selected efficient strains EU-ARP-44, and EU-ARK-23 showed >97% similarity with *Bacillus tropicus* and *B. megaterium*, respectively. The 16S rRNA gene partial sequence was submitted to online NCBI GenBank database and accession number was assigned as ON982713 and ON982714. The strains EU-ARP-44, and EU-ARK-23 were submitted at ICAR-National Bureau of Agriculturally Important Microorganisms (NBAIM) culture-collection facility, Mau Nath Bhanjan, Uttar Pradesh, India. The phylogenetic tree was constructed to know taxonomic affiliation of the potential strains (Figure 1).

**Figure 1:** Phylogenetic tree showing the relationship among nitrogen fixing, phosphorus and potassium solubilizing bacterial isolates, 16S rRNA gene sequences with reference sequences obtained through BLAST analysis. The trees were constructed using neighbor joining (NJ) with algorithm using MEGA 4 software (Tamura et al., 2007).

### 3.4 Evaluation of bacterial consortium

The potential N_2_ fixer (*Rahnella* sp. strain EU-A3SNfb), P-solubilizer (*Bacillus tropicus* EU-ARP-44) and K solubilizer (*B. megaterium* EU-ARK-23) were evaluated as single inoculum and bacterial consortium for PGP of *Aegilops kotschyi* and wheat crop under *in vitro* and *in vivo* conditions.

### 3.5 Evaluation of growth and physiological parameters

The combined effect of PGP bacteria, *Rahnella* sp. strain EU-A3SNfb, *Bacillus tropicus* EU-ARP-44 and *B. megaterium* EU-ARK-23 resulted in growth enhancement of both *Aegilops kotschyi* and wheat crop under *in vitro* and *in vivo* conditions. The growth and physiological parameters of both of the crops were found to be enhanced by the bacterial consortium of EU-A3SNfb, EU-ARP-44, and EU-ARK-23 (Table 1; Table 2). The inoculation of bacterial consortium in *Aegilops kotschyi* and wheat resulted in the increased shoot length by 1.2–1.6 folds under *in vitro* and *in vivo* conditions. The root length of *Aegilops kotschyi* under *in vitro* and *in vivo* were enhanced up to 1.6 and 1.4 fold as compared to control, whereas in wheat bacterial consortium enhanced the length of root by 1.3 fold (*in vitro*) and 1.4 fold (*in vivo*) over control. Bacterial consortium inoculation enhanced the fresh and dry weight of *Aegilops kotschyi* by 2.6 fold and 1.6 fold (*in vitro*); and 4.3 fold and 5.0 fold (*in vivo*) over control, respectively. On the other hand in wheat bacterial consortium incremented the fresh (2.1 and 4.1 fold) and dry weight (2.5 and 3.1 fold) under *in vitro* and *in vivo* conditions in comparison to control, respectively (Figures 2 and 3). The content of chlorophyll is positively affected by the bacterial consortium by 2.2 and 2.0 fold (*Aegilops kotschyi*) and 1.9 and 1.8 fold (wheat) under *in vitro* and *in vivo* conditions as compared to control. Similarly the carotenoids content under *in vitro* and *in vivo* conditions was incremented in *Aegilops kotschyi* (1.4 and 1.5 fold) and wheat (2.1 and 1.5 fold) over control, respectively. The phenolics and flavonoids content were positive affected by the microbial consortium and enhanced up to 3.9 and 2.2 fold in both *Aegilops kotschyi* and wheat over control, respectively. Bacterial consortium enhanced the total soluble sugar content by 1.0 fold (*in vitro*) and 2.6 fold (*in vivo*) in *Aegilops kotschyi* and in wheat was enhanced by 2.4 fold (*in vitro*) and 4.5 fold (*in vivo*) in comparison to control (Figure 4; Figure 5).

RETRACTED

**Table 1:** The effect of the bacterial consortium *Aegilops kotschyi* under *in vivo* conditions.

Treatments	Shoot length (cm)	Root length (cm)	Fresh weight (g)	Dry weight (g)	Chlorophyll (mg/g)	Carotenoids (g/L)	Phenolics (μg/g)	Flavonoid (μg/g)	Soluble sugar (μg/g)
Consortium	53.35^f^ ± 3.16	18.20^e^ ± 2.21	168.25^f^∗ ± 25.93	45.60^e^∗ ± 8.12	26.39^f^ ± 7.46	8.98^e^ ± 0.25	1.00^e^∗ ± 0.02	3.80^f^∗ ± 0.15	55.81^c^ ± 0.80
N-culture	47.45^e^ ± 0.85	15.70^c^ ± 1.50	111.35^e^ ± 34.55	26.90^d^ ± 4.41	16.77^b^ ± 2.57	8.09^d^ ± 0.05	0.90^d^∗ ± 0.00	2.82^c^ ± 0.02	58.00^c^ ± 2.41
P-culture	45.55^d^ ± 0.55	17.35^d^ ± 5.47	94.20^d^ ± 2.11	21.90^c^ ± 1.81	26.08^f^ ± 4.31	7.58^c^ ± 0.98	0.81^c^∗ ± 0.01	3.32^d^∗ ± 0.03	34.67^b^ ± 2.69
K-culture	42.80^c^ ± 2.41	18.00^e^ ± 1.71	77.20^c^ ± 2.81	17.60^c^ ± 3.31	19.82^d^ ± 1.87	8.08^d^ ± 0.69	0.86^c^∗ ± 0.04	2.52^b^ ± 0.00	57.99^c^ ± 1.38
NPK 100%	45.10^d^ ± 1.20	17.40^d^ ± 3.11	65.30^b^ ± 20.26	14.45^b^ ± 4.36	18.47^c^ ± 6.87	5.78^a^ ± 2.13	0.70^b^ ± 0.01	3.43^d^∗ ± 0.22	23.90^a^ ± 1.30
Urea 100%	48.15^e^ ± 8.78	13.6^b^ ± 0.60	102.00^d^ ± 22.37	21.40^c^ ± 1.00	22.06^e^ ± 0.99	8.21^d^ ± 0.25	0.88^d^∗ ± 0.01	2.99^d^∗ ± 0.04	22.18^a^ ± 9.01
DAP 100%	37.95^a^ ± 1.05	18.25^e^ ± 2.16	42.00^a^ ± 0.00	9.10^a^ ± 0.50	17.49^b^ ± 6.25	7.09^b^ ± 0.58	0.42^a^ ± 0.02	3.56^e^∗ ± 0.25	54.12^c^ ± 3.07
Control	41.25^b^ ± 3.96	12.40^a^ ± 0.50	39.60^a^ ± 9.63	9.00^a^ ± 1.60	13.03^a^ ± 0.78	5.74^a^ ± 2.16	0.37^a^ ± 0.25	2.36^a^ ± 0.03	20.99^a^ ± 12.18
LSD	1.18	0.56	10.61	7.92	1.17	0.29	0.05	0.12	4.33
SE	10.94	8.59	58.65	12.52	19.02	4.34	0.21	0.26	20.08
CD 5%	20.73	16.27	111.14	23.72	36.04	8.22	0.40	0.50	38.05

[Numerical values are mean ± Standard deviation of mean (SD) of three independent observations].

RETRACTED

Common superscript code on mean values indicate the non-significant differences among derivatives as based on unpaired Student t-test at p < 0.05. On the other hand, different superscript indicates significant differences among line.

**Table 2:** The effect of the bacterial consortium wheat under *in vivo* conditions.

Treatments	Shoot length (cm)	Root length (cm)	Fresh weight (g)	Dry weight (g)	Chlorophyll (mg/g)	Carotenoids (g/L)	Phenolics (μg/g)	Flavonoid (μg/g)	Soluble sugar (μg/g)
Consortium	111.33^d^∗ ± 2.34	14.13^d^ ± 1.96	146.10^h^∗ ± 7.20	46.50^h^∗ ± 11.65	39.23^d^∗ ± 8.15	6.98^c^ ± 0.86	2.04^f^ ± 0.08	7.28^e^ ± 0.64	37.94^g^∗ ± 0.04
N-culture	111.20^d^∗ ± 0.51	15.57^e^ ± 2.03	129.90^g^∗ ± 32.55	43.77^g^∗ ± 2.85	29.24^c^ ± 0.53	4.94^a^ ± 0.09	1.47^d^ ± 0.06	5.53^b^ ± 0.61	17.11^c^ ± 1.79
P-culture	103.80^c^∗ ± 2.75	12.87^c^ ± 0.63	105.37^f^∗ ± 2.46	34.40^e^∗ ± 2.16	23.61^b^ ± 9.54	6.16^b^ ± 0.44	1.57^e^ ± 0.08	6.81^d^ ± 0.71	12.79^b^ ± 0.05
K-culture	112.37^d^∗ ± 2.04	12.20^b^ ± 0.50	80.93^d^ ± 0.72	27.57^d^∗ ± 1.69	27.36^c^ ± 2.65	4.74^a^ ± 0.09	1.54^d^ ± 0.05	5.56^b^ ± 0.61	28.58^f^∗ ± 4.36
NPK 100%	96.40^b^ ± 3.76	11.90^b^ ± 0.26	67.40^b^ ± 5.64	22.20^b^∗ ± 3.17	29.16^c^ ± 8.44	6.08^b^ ± 1.15	1.13^a^ ± 0.06	5.87^c^ ± 0.96	21.68^e^∗ ± 4.39
Urea 100%	99.87^c^ ± 0.77	13.63^d^ ± 0.67	89.47^e^∗ ± 13.83	42.30^f^∗ ± 7.32	22.17^a^ ± 1.81	5.60^b^ ± 0.08	1.35^c^ ± 0.06	6.96^d^ ± 0.27	18.89^d^∗ ± 1.20
DAP 100%	110.03^d^∗±5.64	14.10^d^ ± 2.06	76.43^c^ ± 11.04	25.80^c^∗±2.45	24.39^b^ ± 4.84	4.81^a^ ± 0.12	1.21^b^ ± 0.23	7.39^e^ ± 1.17	15.31^c^ ± 5.53
Control	85.27^a^ ± 4.75	9.57^a^ ± 0.35	35.27^a^ ± 1.99	14.80^a^ ± 3.08	20.87^a^ ± 0.30	4.60^a^ ± 0.83	1.13^a^ ± 0.23	4.43^a^ ± 0.36	8.48^a^ ± 1.07
LSD	2.79	0.69	3.86	0.55	2.20	0.65	0.07	0.30	1.86
SE	8.43	4.15	24.77	3.86	7.98	1.56	0.53	2.65	5.20
CD 5%	15.98	7.86	46.94	7.31	15.12	2.96	1.00	5.03	9.86

[Numerical values are mean ± Standard deviation of mean (SD) of three independent observations].

RETRACTED

Common superscript code on mean values indicate the non-significant differences among derivatives as based on unpaired Student t-test at p < 0.05. On the other hand, different superscript indicates significant differences among line.

**Figure 2:** Effect of the bacterial consortium on the growth parameters of *Aegilops kotschyi*. Bacterial consortium: *Rahnella* sp. strain EU-A3SNfb, *Bacillus tropicus* EU-ARP-44, and *B. megaterium* EU-ARK-23; EU-A3SNfb: *Rahnella* sp. strain EU-A3SNfb (Nitrogen fixer); EU-ARP-44: *Bacillus tropicus* EU-ARP-44 (Phosphorus solubilizer); EU-ARK-23: *B. megaterium* EU-ARK-23 (Potassium solubilizer); DAP: Di-ammonium phosphate. [Common superscript code on mean values indicate the non-significant differences among derivatives as based on unpaired Student t-test at p < 0.05. On the other hand, different superscript indicates significant differences among lines].

**Figure 3:** Effect of the bacterial consortium on the growth parameters of wheat. Bacterial consortium: *Rahnella* sp. strain EU-A3SNfb, *Bacillus tropicus* EU-ARP-44, and *B. megaterium* EU-ARK-23; EU-A3SNfb: *Rahnella* sp. strain EU-A3SNfb (Nitrogen fixer); EU-ARP-44: *Bacillus tropicus* EU-ARP-44 (Phosphorus solubilizer); EU-ARK-23: *B. megaterium* EU-ARK-23 (Potassium solubilizer); DAP: Di-ammonium phosphate. [Common superscript code on mean values indicate the non-significant differences among derivatives as based on unpaired Student t-test at p < 0.05. On the other hand, different superscript indicates significant differences among lines].

**Figure 4:** a. Effect of bacterial consortium on chlorophyll content of *Aegilops kotschyi.* Bacterial consortium: *Rahnella* sp. strain EU-A3SNfb, *Bacillus tropicus* EU-ARP-44, and *B. megaterium* EU-ARK-23; EU-A3SNfb: *Rahnella* sp. strain EU-A3SNfb (Nitrogen fixer); EU-ARP-44: *Bacillus tropicus* EU-ARP-44 (Phosphorus solubilizer); EU-ARK-23: *B. megaterium* EU-ARK-23 (Potassium solubilizer); DAP: Di-ammonium phosphate. [Common superscript code on mean values indicate the non-significant differences among derivatives as based on unpaired Student t-test at p < 0.05. On the other hand, different superscript indicates significant differences among lines]. b. Effect of bacterial consortium on carotenoids content of *Aegilops kotschyi.* Bacterial consortium: *Rahnella* sp. strain EU-A3SNfb, *Bacillus tropicus* EU-ARP-44, and *B. megaterium* EU-ARK-23; EU-A3SNfb: *Rahnella* sp. strain EU-A3SNfb (Nitrogen fixer); EU-ARP-44: *Bacillus tropicus* EU-ARP-44 (Phosphorus solubilizer); EU-ARK-23: *B. megaterium* EU-ARK-23 (Potassium solubilizer); DAP: Di-ammonium phosphate. [Common superscript code on mean values indicate the non-significant differences among derivatives as based on unpaired Student t-test at p < 0.05. On the other hand, different superscript indicates significant differences among lines]. c. Effect of bacterial consortium on phenolic content of *Aegilops kotschyi*. Bacterial consortium: *Rahnella* sp. strain EU-A3SNfb, *Bacillus tropicus* EU-ARP-44, and *B. megaterium* EU-ARK-23; EU-A3SNfb: *Rahnella* sp. strain EU-A3SNfb (Nitrogen fixer); EU-ARP-44: *Bacillus tropicus* EU-ARP-44 (Phosphorus solubilizer); EU-ARK-23: *B. megaterium* EU-ARK-23 (Potassium solubilizer); DAP: Di-ammonium phosphate. [Common superscript code on mean values indicate the non-significant differences among derivatives as based on unpaired Student t-test at p < 0.05. On the other hand, different superscript indicates significant differences among lines]. d. Effect of bacterial consortium on flavonoid content of *Aegilops kotschyi*. Bacterial consortium: *Rahnella* sp. strain EU-A3SNfb, *Bacillus tropicus* EU-ARP-44, and *B. megaterium* EU-ARK-23; EU-A3SNfb: *Rahnella* sp. strain EU-A3SNfb (Nitrogen fixer); EU-ARP-44: *Bacillus tropicus* EU-ARP-44 (Phosphorus solubilizer); EU-ARK-23: *B. megaterium* EU-ARK-23 (Potassium solubilizer); DAP: Di-ammonium phosphate. [Common superscript code on mean values indicate the non-significant differences among derivatives as based on unpaired Student t-test at p < 0.05. On the other hand, different superscript indicates significant differences among lines]. e. Effect of bacterial consortium on soluble sugar content of *Aegilops kotschyi*. Bacterial consortium: *Rahnella* sp. strain EU-A3SNfb, *Bacillus tropicus* EU-ARP-44, and *B. megaterium* EU-ARK-23; EU-A3SNfb: *Rahnella* sp. strain EU-A3SNfb (Nitrogen fixer); EU-ARP-44: *Bacillus tropicus* EU-ARP-44 (Phosphorus solubilizer); EU-ARK-23: *B. megaterium* EU-ARK-23 (Potassium solubilizer); DAP: Di-ammonium phosphate. [Common superscript code on mean values indicate the non-significant differences among derivatives as based on unpaired Student t-test at p < 0.05. On the other hand, different superscript indicates significant differences among lines].

RETRACTED

**Figure 5:** a. Effect of bacterial consortium on chlorophyll content of wheat. Bacterial consortium: *Rahnella* sp. strain EU-A3SNfb, *Bacillus tropicus* EU-ARP-44, and *B. megaterium* EU-ARK-23; EU-A3SNfb: *Rahnella* sp. strain EU-A3SNfb (Nitrogen fixer); EU-ARP-44: *Bacillus tropicus* EU-ARP-44 (Phosphorus solubilizer); EU-ARK-23: *B. megaterium* EU-ARK-23 (Potassium solubilizer); DAP: Di-ammonium phosphate. [Common superscript code on mean values indicate the non-significant differences among derivatives as based on unpaired Student t-test at p < 0.05. On the other hand, different superscript indicates significant differences among lines]. b. Effect of bacterial consortium on carotenoids content of wheat. Bacterial consortium: *Rahnella* sp. strain EU-A3SNfb, *Bacillus tropicus* EU-ARP-44, and *B. megaterium* EU-ARK-23; EU-A3SNfb: *Rahnella* sp. strain EU-A3SNfb (Nitrogen fixer); EU-ARP-44: *Bacillus tropicus* EU-ARP-44 (Phosphorus solubilizer); EU-ARK-23: *B. megaterium* EU-ARK-23 (Potassium solubilizer); DAP: Di-ammonium phosphate. [Common superscript code on mean values indicate the non-significant differences among derivatives as based on unpaired Student t-test at p < 0.05. On the other hand, different superscript indicates significant differences among lines]. c. Effect of bacterial consortium on phenolic content of wheat. Bacterial consortium: *Rahnella* sp. strain EU-A3SNfb, *Bacillus tropicus* EU-ARP-44, and *B. megaterium* EU-ARK-23; EU-A3SNfb: *Rahnella* sp. strain EU-A3SNfb (Nitrogen fixer); EU-ARP-44: *Bacillus tropicus* EU-ARP-44 (Phosphorus solubilizer); EU-ARK-23: *B. megaterium* EU-ARK-23 (Potassium solubilizer); DAP: Di-ammonium phosphate. [Common superscript code on mean values indicate the non-significant differences among derivatives as based on unpaired Student t-test at p < 0.05. On the other hand, different superscript indicates significant differences among lines]. d. Effect of bacterial consortium on flavonoid content of wheat. Bacterial consortium: *Rahnella* sp. strain EU-A3SNfb, *Bacillus tropicus* EU-ARP-44, and *B. megaterium* EU-ARK-23; EU-A3SNfb: *Rahnella* sp. strain EU-A3SNfb (Nitrogen fixer); EU-ARP-44: *Bacillus tropicus* EU-ARP-44 (Phosphorus solubilizer); EU-ARK-23: *B. megaterium* EU-ARK-23 (Potassium solubilizer); DAP: Di-ammonium phosphate. [Common superscript code on mean values indicate the non-significant differences among derivatives as based on unpaired Student t-test at p < 0.05. On the other hand, different superscript indicates significant differences among lines]. e. Effect of bacterial consortium on soluble sugar content of wheat. Bacterial consortium: *Rahnella* sp. strain EU-A3SNfb, *Bacillus tropicus* EU-ARP-44, and *B. megaterium* EU-ARK-23; EU-A3SNfb: *Rahnella* sp. strain EU-A3SNfb (Nitrogen fixer); EU-ARP-44: *Bacillus tropicus* EU-ARP-44 (Phosphorus solubilizer); EU-ARK-23: *B. megaterium* EU-ARK-23 (Potassium solubilizer); DAP: Di-ammonium phosphate. [Common superscript code on mean values indicate the non-significant differences among derivatives as based on unpaired Student t-test at p < 0.05. On the other hand, different superscript indicates significant differences among lines].

RETRACTED

## 4 Discussion

Bacteria can boost the availability of nutrient for plant through fixing nitrogen, solubilizing inorganic phosphorus, potassium, zinc and producing of siderophores (Patni et al., 2018). The bacterial strains also protect plant from pest and pathogen by producing cellulose, pectinase, xylanase, amylase, and gelatinase (Glick 2012). In the present study total of 125 endophytic and rhizospheric bacteria were isolated from *Aegilops kotschyi*. The fact that Nitrogen (N) is component of protein, nucleic acid and the cells energy currency, make it a vital macronutrient that is absolutely necessary for plant growth and productivity (Rana et al., 2020). Despite nitrogen consists nearly 80% in our atmosphere, most life forms cannot utilize it because of its inert state (Doty 2017a). Endophytic microorganism can fix more nitrogen even better than rhizosphere microbes because nitrogen fixation in plant interior is suitable due to low partial oxygen pressure (James and Olivares 1998). In the present study, *Rahnella* sp. EU-A3SNfb a promising nitrogen-fixing bacterium isolated previously from *Aegilops kotschyi* have maximal nitrogenase activity of 25.02 ± 0.09 nmol C_2_H_4_ mg^−1^ protein hr^−1^ (Negi et al., 2022). In a another report, *Rahnella* sp. GT24B from *Valeriana pycnantha* and *Gentianella weberbaueri* wild medicinal Peruvian plants was reported as solubilizer of inorganic phosphate and produces siderophores (Ulloa-Muñoz et al., 2020).

Phosphorus (P) is a necessary element that is categorized as a macronutrient because it is required in higher amounts by the plant for proper growth. It could be found in soil in the form of mineral salts or combined with organic compounds (Kour et al., 2021). Despite the fact that total phosphate is usually abundant in agricultural soils, most of them exist in an insoluble forms that cannot be absorbed by plant (Miller et al., 2010). The optimum productivity, plant need nearly 30 mol L^−1^ of phosphorus, but only about 1 mol L^−1^ of phosphorus is present in much soil. As a result, it has been noted that phosphorus unavailability in many soils is a significant growth limitation in agricultural production systems (Daniels et al., 2009). The only strategies used currently to maintain and increase agricultural and horticultural productivity are chemical fertilizers and insecticides (Jabborova et al., 2021). Even through the use of chemical fertilizers increase the agricultural production of about 50%, they are also closely linked to environmental damage and health issues in both humans and animals (Walia et al., 2017). In a present investigation, Pikovskaya agar was used to examine the phosphate solubilization capacity of rhizospheric bacteria. The result showed that *Bacillus tropicus* EU-ARP-44 isolated from goatgrass rhizosphere was showed maximum phosphorus solubilizing activity of 270.5 ± 0.00 mg L^−1^. In a similar finding Mir et al. (2021) *Pseudomonas aeruginosa* and *Enterobacter* sp. IHK-3 were isolated from rice and these bacteria have ability to solubilize inorganic phosphorus ranging from 312.4 ± 1.15 and 298.7 ± 1.25 μg mL^−1^). These bacterial IHK-3 and IHK-25 also produce siderophores, HCN and ammonia. In an investigation, *Bacillus tropicus* ZA1 was isolated from rhizospheric region and it was able to solubilizes inorganic phosphate, produce IAA and siderophores (Nandal and Solanki 2021). Jaya et al. (2019) reported, *Bacillus tropicus* was isolated from rhizosphere of pineapple.

RETRACTED

After N and P, potassium ranks as the third-most significant primary necessary plant nutrient. It plays a critical part in the metabolism of plants by activating the most significant enzymes involved in their physiology. Potassium insufficiency affects with plant physiology, impairing growth and leads to lower yields (White and Karley 2010). Potassium is found in the soil as an insoluble K mineral, which cannot easily utilized by plant. In soil there are certain microbes present that can be employed to boost K availability from soil to plant are known as potassium solubilizing microbes (Kaur et al., 2021). The over use of chemical fertilizer has negative effect on ecosystem which can be decrease by using phosphorus, potassium solubilizing microorganism in agriculture which can contribute for making sustainable agriculture (Suyal et al., 2021). In present study *Bacillus megaterium* EU-ARK-23 was isolated from rhizosphere of goatgrass have ability to solubilize potassium. In a report, *Bacillus megaterium* BHU1 was isolated from rhizospheric soil and it was reported for producing ammonia and solubilizing maximum amount phosphorus after 2 and 5 days ranging from 121.2 and 153.6 mg ml⁻^1^ as compared to uninoculated control (Kumar et al., 2014). In another report *Bacillus megaterium* TRS-4 was isolated from rhizospheric region of tea and this strain promotes the plant growth by phosphorus solubilization, production IAA siderophores and antifungal metabolite (Chakraborty et al., 2006). Chandra et al. (2018) reported, *Bacillus megaterium* BMSE7 from rhizospheric region of sugarcane. The treated sugarcane seed with culture of *Bacillus megaterium* was resulted in the significant increment in fresh/dry weight, and chlorophyll content. In a report, *Pseudomonas fragi* (EPS 1) significantly increase the root dry weight and zinc content in wheat (Kamran et al., 2017). Mena-Violante and Olalde-Portugal (2007) reported, inoculation of *Bacillus subtilis* BEB-13bs increase dry weight and length of root of tomato plants.

RETRACTED

The combine application of N-fixing (*Rahnella* sp. strain EU-A3SNfb), P-solubilizing (*Bacillus tropicus* EU-ARP-44) and K solubilizing (*B. megaterium* EU-ARK-23) strains shown to increment the chlorophyll and carotenoids content in *Aegilops kotschyi* and wheat plants both *in vitro* and *in vivo*. Triple combination of compatible rhizosphere microbes *Mesorhizobium* sp. (RL091), *Pseudomonas aeruginosa* (PHU094), and *Trichoderma harzianum* (THU0816) promote higher growth in chickpea as compared to untreated control (Singh et al., 2014). Devi et al. (2022b) reported, the microbial consortium of *Erwinia rhapontici* EU-B1SP1, *Bacillus* sp. strains IARI-HHS2-45, and *Pseudomanas gessardi* EU-LWNA-25 significantly increases the growth as well as physiological parameters of *Amaranthus* plants as compared to untreated control. In another study Choure and Dubey (2012), inoculated the combined mixture of *Azotobacter chroococcum* AZK2, *Pseudomonas fluorescens* LPK2, and *Sinorhizobium fredii* KCC5 in *Cajanus cajan* and maximum plant growth of as compared to control was observed. The combined mixture of bacterial strain LPK2, KCC5and AZK2 increased seed germination and enhanced early growth of *Cajanus cajan.* The combined inoculation of *B. megaterium, A. chlorophenolicus and Enterobacter* showed significant increment in plant height, acquisition of nitrogen and phosphorus in grain as compared to untreated control (Kumar et al., 2014). In a similar finding microbial inoculation of *Pseudomonas putida*, *Glomus intraradices, Bacillus polymixa*, and *Azotobacter chroococcum* showed significant enhancement of chlorophyll and NPK content in plant and also incremented the root and shoot biomass (Vafadar et al., 2014). In a present study, the microbial mixture inoculation showed significant increment in carotenoids content and sugar content in wheat. Inoculation of microbial mixture of two salt-tolerant bacteria *Aneurinibacillus aneurinilyticus* AIOA1 and *Paenibacillus* sp. SG_AIOA2 significantly incremented chlorophyll, carotenoids, total soluble sugar and proline content, along with biomass of root/shoot and length of common bean plants (Gupta and Pandey 2020). The content of phenolic and flavonoids have been reported to be enhanced by microbial mixture of *Rahnella* sp. EU-A_3_SNfb, *Bacillus tropicus* EU-ARP-44 and *Bacillus megaterium* EU-ARK-23 in the present study. In a report, microbial mixture of *Bacillus subtilis, Pseudomonas aeruginosa* and *Trichoderma harzianum* showed enhancement in total phenolic and flavonoid content in pea plant (Jain et al., 2014).

RETRACTED

In conclusion, the bacterial consortium of N-fixer (*Rahnella* sp. strain EU-A3SNfb), P-solubilizer (*Bacillus tropicus* EU-ARP-44) and K solubilizer (*B. megaterium* EU-ARK-23) incremented the growth of the wheat and wild wheat relative *Aegilops kotschyi* more with respect to individual inoculation of bacterial, different chemicals and untreated control. In best of our knowledge, this is first ever report that has reported the development of bacterial consortium from the bacteria associated with wild wheat relative *Aegilops kotschyi*. In recent times, reduction of agrochemical is an emergence for agricultural and environmental sustainability, thus the use of bacterial consortium as bioinoculant could be an appropriate biofertilizer for cereal crops. In future the bacterial consortium could be evaluated on the diverse horticultural and cereal crops. The strains could be genetically modified through the genetic manipulation for better performance to improve the crop productivity.

## Declarations

### Author contribution statement

Rajeshwari Negi; Tanvir Kaur; Rubee Devi: Performed the experiments; Analyzed and interpreted the data; Wrote the paper.

Divjot Kour: Contributed reagents, materials, analysis tools or data.

Ajar Nath Yadav: Conceived and designed the experiments.

### Funding statement

This research did not receive any specific grant from funding agencies in the public, commercial, or not-for-profit sectors.

### Data availability statement

No data was used for the research described in the article.

### Declaration of interest’s statement

The authors declare no competing interests.

### Additional information

No additional information is available for this paper.
